This article has been retracted.

# Effect and Potential Mechanism of *Lactobacillus plantarum* Q7 on Hyperuricemia *in vitro* and *in vivo*

**DOI:** 10.3389/fnut.2022.954545

**Published:** 2022-07-06

**Authors:** Jiayuan Cao, Yushan Bu, Haining Hao, Qiqi Liu, Ting Wang, Yisuo Liu, Huaxi Yi

**Affiliations:** College of Food Science and Engineering, Ocean University of China, Qingdao, China

**Keywords:** Hyperuricemia, *Lactobacillus plantarum* Q7, uric acid, gut microbiota, inflammatory cytokines

## Abstract

Hyperuricemia (HUA) is a disorder of purine metabolism resulting in abnormally elevated serum uric acid (UA) concentration. It is believed that there is an association between gut microbiota and HUA, and probiotics have the potential palliative effect. However, the underlying mechanism of probiotics in ameliorating HUA remains unclear. The purpose of this study was to investigate the effect and mechanism of *Lactobacillus plantarum* Q7 on HUA in Balb/c mice. The results showed that *L. plantarum* Q7 had an excellent capability to affect UA metabolism, which could degrade nucleotides by 99.97%, nucleosides by 99.15%, purine by 87.35%, and UA by 81.30%. It was observed that *L. plantarum* Q7 could downregulate serum UA, blood urea nitrogen (BUN), creatinine (Cr), and xanthine oxidase (XOD) by 47.24%, 14.59%, 54.59%, and 40.80%, respectively. Oral administration of *L. plantarum* Q7 could restore the liver, kidney, and intestinal injury induced by HUA and the expression of metabolic enzymes and transporters to normal level. 16S rRNA sequencing analysis showed that *L. plantarum* Q7 treatment could restore the imbalance of species diversity, richness, and community evenness compared with the model group. The ratio of *Bacteroidetes* to *Firmicutes* was recovered nearly to the normal level by *L. plantarum* Q7 intervention. The dominant microorganisms of *L. plantarum* Q7 group contained more anti-inflammatory bacteria than those of the model group. These findings indicated that *L. plantarum* Q7 might regulate UA metabolism and repair the liver and kidney injury by reshaping the gut microbiota and could be used as a potential probiotic strain to ameliorate HUA.

## Introduction

Hyperuricemia (HUA) is a metabolic syndrome characterized by the persistently elevated serum uric acid (UA) concentration above 7 mg/dl in men and 6 mg/dl in women (1). It is a major risk factor for the progression of high comorbidity burden and finally leads to tissue damage, such as gout (2), type 2 diabetes mellitus (3), atherosclerosis (4), and chronic nephrosis (5). In addition, it has been shown that HUA was common in patients with advanced chronic systolic heart failure and HUA increased their hospitalization and mortality (6). Globally, the incidence of HUA shows a trend of rapid increase by about 20% (7–9). HUA has been considered as the fourth-highest risk factor after hyperlipidemia, hypertension, and hyperglycemia (10). Although there are some drugs or dietary therapy to reduce serum UA, some side effects, such as the associated risk of kidney stone and all-cause cardiac death, prevent patients from making long-term choices (11). Overall, it is significant to develop an effective and safe treatment for HUA.

Uric acid is the final product of purine metabolism in the human body (2), which is regulated by the metabolism of liver, kidney, and intestine (12). Since there is no uricase to convert urate to the water-soluble allantoin in the human body (13), the UA level is easily influenced if there is a disorder of UA purine metabolism (14). The excretion of UA is regulated by the kidney and intestine, and about 30% of UA is excreted and metabolized by gut bacteria (15). Emerging evidence shows that ecological dysbiosis of intestinal flora is inextricably linked to the development of many metabolic diseases (16). It was found that *Bacteroides caccae* and *Bacteroides xylanisolvens* were rich in the HUA patients, while *Faecalibacterium prausnitzii* and *Bidobacterium pseudocatenulatum* were significantly absent (17). Thus, the regulation of gut microbiota has become a new target for alleviating HUA (18). It was reported that probiotics could alleviate HUA by maintaining normal gut microbiota, enhancing mucosal barrier function, and inhibiting exposure to inflammatory signals, which are expected to be a new treatment for HUA (19–21).

In our previous study, *L. plantarum* Q7 was isolated from the traditional Chinese fermented foods (22) and was observed to exhibit antibacterial activity against pathogenic bacteria associated with ulcerative colitis (23). In this study, the effect of *L. plantarum* Q7 on UA metabolism and excretion in an HUA mice model was evaluated, which might provide a basis for the development of probiotics to alleviate HUA.

## Materials and Methods

### Cultivation of *L. plantarum* Q7

*Lactobacillus plantarum* Q7 (GenBank: CP019712-16) was isolated from traditional fermented yak yogurt in Qinghai Province, China (24); 2% (v/v) *L. plantarum* Q7 was inoculated in de Man, Rogosa, and Sharpe (MRS) liquid medium (Hopebio Technology, Qingdao, China) and cultured at 37°C for 24 h. OD was measured at 600 nm to evaluate the growth state of *L. plantarum* Q7.

### Determination of UA Degradation Activity of *L. plantarum* Q7 *in vitro*

Fermentation broth of the activated *L. plantarum* Q7 was centrifuged at 8,000 rpm for 10 min at 4°C. The sediments of bacterial cells were washed two times with sterile phosphate-buffered saline (PBS) and suspended again in 1 ml nucleotide-neutral potassium phosphate solution, nucleoside-neutral potassium phosphate solution, purine-neutral potassium phosphate solution, uric-neutral potassium phosphate solution (100 mmol/L, pH = 7), respectively. The concentration of *L. plantarum* Q7 was determined to be 10^9^ CFU/ml by the plate counting method (25). The mixed solution was incubated in AnaeroPack (Mitsubishi Gas Chemical Co., Inc., Tokyo, Japan) at 37°C to obtain anaerobic condition. After incubation for 30 min, the mixture was mixed with perchloric acid as a terminator and filtered through a 0.22 μm filter. Then, 20 μl mixed solution was extracted and analyzed by HPLC (Shimadzu, Tokyo, Japan) (Chromatographic column: ZORBAX Eclipse Plus C18, 4.6 × 250 mm, 5-Micron; UV detection wavelength: 254 nm; Mobile phase: 20 mmol/L isogradient phosphate-buffered solution; Flow rate: 1 ml/min; Elution time: 45 min; Column temperature: 25°C). Corresponding results were calculated by the following formula (20):


$$\text{Degradation}\;\text{rate}\;(\text{\%})\;=\;\frac{\left({\text{C}}_{\text{Standard}}-{\text{C}}_{\text{Sample}}\right)}{{\text{C}}_{\text{Standard}}}\;*\;100\text{\%}$$

### Probiotic Properties Assay of *L. plantarum* Q7

The resistance of *L. plantarum* Q7 to acid, bile salts, and simulated gastrointestinal juices was determined according to the previous report (26) with minor modifications. The overnight cultured *L. plantarum* Q7 was centrifuged at 6,000 rpm for 10 min at 4°C, and then, the sediments of bacterial cells were washed two times with PBS. The cells of *L. plantarum* Q7 were resuspended and cultured in MRS (adjusted to pH 3.0) for 3 h, MRS supplemented with 0.3% bile salts for 5 h, simulated gastric juice for 3 h, and simulated intestinal juice for 8 h, respectively. The bacterial survival rate was assayed by the plate colony counting method and calculated according to the following equation (26):


$$\begin{array}{l} \text{Survival}\;\text{rate}\;(\text{\%})\\ \;=\frac{\text{logCFUtotal}\;\text{viable}\;\text{counts}\;\text{after}\;\text{treatment}}{\text{logCFUtotal}\;\text{viable}\;\text{counts}\;\text{before}\;\text{treatment}}\;*\;100\text{\%} \end{array}$$

### Treatment of Animals

Six-week-old specific-pathogen-free (SPF) male Balb/c mice were purchased from Beijing Weitong Lihua Experimental Animal Technology Co., Ltd. [Animal Qualification Certificate Number: SCXK (Beijing) 2014-0001]. Mice were acclimatized in an animal care facility with 12 h light/dark cycles and 50%−70% relative humidity at 18–24°C. Sufficient food (Beijing Keao Xieli Feed Co., Ltd., Beijing, China) and water were provided. All experimental processes were approved by the Animal Ethics Committee of Ocean University of China (Permission number: SPXY2022011201).

### Model Establishment of HUA Mice

The mice were randomly divided into four groups according to their initial weight, namely, control group (CON), model group (MOD), probiotics group (Q7), and active drug control group (ADC). For the entire duration of the experiment, the CON group was fed a normal diet and water, while the other groups were fed a high-purine diet (containing 400 g/kg yeast extract and 20 g/kg ribonucleic acid from torula yeast) and 5% fructose water. To induce HUA, the mice in the MOD group were intraperitoneally injected with potassium oxazinate solution (400 mg/kg in 0.5% CMC-NA), and the mice in the CON group were injected with 0.5% CMC-NA for 4 weeks.

After 2-week modeling, gavaging of 10 ml/kg was started. The CON group and the MOD group were given 0.85% NaCl, the Q7 group was given 10^9^ CFU/ml of *L. plantarum* Q7 in 0.85% NaCl, and the ADC group was given 42 mg/kg of allopurinol (ALLO) in 0.85% NaCl. The specific establishment and treatment period of the HUA model are shown in Figure 1.

**Figure 1:** Experimental chart in the treatment of HUA mice.

### Measurement of Body Weight and Organ Co-efficient

Body weight of mice was recorded every week, and weight changes in the different groups were monitored. The whole kidney weight and the liver weight were measured, and the organ index of mice was calculated according to the following formula in a recent report (25).


$$\text{Organ}\;\text{index}\;(\text{\%})\;=\;\frac{{\text{M}}_{\text{Organ}}}{{\text{M}}_{\text{Body}}}*100\text{\%}$$

### Assay of Serum Biochemical Indexes

Blood samples were collected from the eyeball veins of mice on the 7th, 21st, and 35th day. Then, they were placed for 2 h and centrifuged to obtain the supernatant. The serum biochemical indexes of uric acid (UA), blood urea nitrogen (BUN), creatinine (Cr), and xanthine oxidase (XOD) were measured with ELISA kits (Kaerwen, Suzhou, China) according to the manuscript's protocol.

### Analysis of Histophysiology

Liver, kidney, and intestinal tissues of mice were collected and stored in a refrigerator at −80°C. According to a previous method (19), 0.8 × 0.8 cm mice liver and kidney fan-shaped tissue samples and 1 cm mice ileum tissue were fixed in 4% paraformaldehyde for 24 h and then embedded in paraffin. One piece was cut from the paraffin block (4 μm thick), and H&E-stained samples were observed and photographed under an optical microscope (Nikon, Tokyo, Japan).

### Detection of Inflammation Cytokines Levels

Hepatic and renal tissue samples were homogenized in 0.9% cold saline at 60 Hz for 1 min by a tissue grinder (Servicebio, Wuhan, China) and then centrifuged at 5,000 rpm for 10 min to obtain the supernatant. The levels of tumor necrosis factor-α (TNF-α), interleukin-1β (IL-1β), and malondialdehyde (MDA) in homogenate and the concentration of IL-1β and lipopolysaccharide (LPS) in the serum were determined using ELISA kits (Kaerwen, Suzhou, China) according to the manufacturer's instructions.

### Determination of Hepatic Metabolism Enzyme

The hepatic tissue was processed by a tissue grinder according to the method described in the “Detection of inflammation cytokines levels” section. Response of metabolic enzymes, such as adenosine deaminase (ADA) and xanthine oxidase (XOD), in the liver were determined by the ELISA kit (Kaerwen, Suzhou, China) according to the instructions.

### Assay of UA Metabolism Transporters Expression by Real-Time PCR

The nephritic tissue was put into 1 ml TRIzol reagent (Biosharp, Beijing, China) and homogenized as described in the “Detection of inflammation cytokines levels” section. The mRNA was reverse transcribed *via* a high-capacity cDNA using the 5 × All-In-One RT MasterMix reverse transcription reaction kit (ABM, Vancouver, Canada). The gene primer sequences of urate transporter 1 (URAT1), glucose transporter 9 (GLUT9), and sodium-phosphate cotransporter type 1 (NPT1) were synthesized by Sangon Biotech Co., Ltd. (Shanghai, China) (Table 1). Genes were quantitated *via* real-time PCR instrument (ABI, Massachusetts, USA). Changes in mRNA expression were calculated as a relative fold change.

**Table 1:** Target gene primer sequences.

**Gene**	**Forward (5′-3′)**	**Reverse (5′-3′)**
β-actin	ACTGCTCTGGCTCCTAGCAC	CCACCGATCCACACAGAGTA
GLUT9	ATGTGGACTCAATGCGATCTGGTTC	TGTTTCAATTCCTCCCGTGCTCAG
NPT1	TGTTGGGTGTGTTCTGAGTCTTTCC	CCTTCTCACTGCTGCTCATATACGG
URAT1	GACCTTGGACCCGATGTTCTTCTG	CGTGGCGTTGGACTCTGTAAGC

### 16S rRNA Gene Sequencing of Gut Microbiota

The feces were collected from individually housed mice on the last day of intragastric treatment and immediately frozen at −80°C until DNA extraction. The fecal genomic DNA extraction was performed by the Fast DNA SPIN extraction kit (MP Biomedicals, Santa Ana, USA), and then it was amplified through high-throughput sequencing using a Q5 High Fidelity DNA Polymerase. The highly variable V3–V4 regions were amplified using the forward primer 338F (ACTCCTACGGGAGGCAGCA) and the reverse primer 806R (TCGGACTACHVGGGTWTCTAAT). 16S rRNA gene sequencing was conducted by Shanghai Personal Biotechnology Co., Ltd. (Shanghai, China).

### Statistical Analyses

All data were expressed as the mean ± SD, and all analyses were performed in triplicate. The experimental data were analyzed by the GraphPad Prism version 7.0 and SPSS 25.0 statistical software.

## Results and Discussion

### UA-Lowering Activity and Gastrointestinal Tolerance of *L. plantarum* Q7 *in vitro*

The production and excretion of UA are complex processes involving purine metabolism, as well as renal and gut excretion. Two-thirds of UA is eliminated by the kidneys, and one-third of UA is eliminated by the gastrointestinal tract. It suggested that regulating purine metabolism or gut microbiota might be a potential strategy to keep the balance of UA. In our preliminary experiment, it was found that *L. plantarum* Q7 from Chinese traditional food had the ability to reduce UA. In this study, the effect of *L. plantarum* Q7 on the substances associated with purine metabolism was further measured. The assimilating abilities of nucleotide, nucleoside, purine, and UA were evaluated based on HPLC. Results were shown in Figure 2A, and it was observed that *L. plantarum* Q7 could degrade nucleotides by 99.97%, nucleosides by 99.15%, purine by 87.35%, and UA by 81.30% (*P* < 0.05), respectively. It indicated that *L. plantarum* Q7 might exhibit UA-lowering activity by regulating UA production and degradation. Wu et al. (21) reported that *Limosilactobacillus fermentum* JL-3 could ameliorate HUA by degrading UA. In addition, it has been reported that the gut microbiota could be a target to control HUA (17, 27), which is gaining much attention to regulate the whole process of UA metabolism through probiotic intestinal therapy (19–21). Compared with the existing reports, *L. plantarum* Q7 showed a stronger comprehensive assimilation ability to regulate UA metabolism.

**Figure 2:** Determination of UA-lowering activity and gastrointestinal tolerance of L. plantarum Q7. **(A)** UA-lowering activity; **(B)** Gastrointestinal tolerance.

The tolerance to acid, bile salt, and the gastrointestinal tract is the prerequisite for probiotics to exert function *in vivo*. The tolerance of *L. plantarum* Q7 to acid, bile salts, and simulated gastrointestinal juices was determined and is shown in Figure 2B. It was shown that the survival rate of *L. plantarum* Q7 under the above conditions could reach 93.43%, 80.05%, 93.97%, and 99.02% (*P* < 0.05), respectively. The results suggested that *L. plantarum* Q7 had excellent tolerance to the harsh gastrointestinal environment.

### Alleviation of HUA Symptom in Mice by *L. plantarum* Q7

The common experimental animals, such as mice, can express urate oxidase, which catalyzes the oxidation of UA to hydrogen peroxide, carbon dioxide, and allantoin in most mammals (28). However, urate oxidase is lost during the human revolution by some unknown mutation. To induce the state of HUA, potassium oxyazinate intraperitoneal injection combined with high-purine food and fructose water was selected. The effect of *L. plantarum* Q7 on HUA was evaluated in Balb/c mice. The body weight, organ weight, visceral Co-efficient, and viscus histomorphology were analyzed first. As shown in Table 2, there was no statistical difference in the weight of mice after adaptation. However, the body weight of mice in the CON and Q7 groups was significantly higher than that of the MOD and ADC groups (*P* < 0.05) at the end of the experiment. Compared with the MOD group, the weight loss could be slowed by *L. plantarum* Q7 intervention. Similarly, the organ weight and the visceral Co-efficient of the MOD group were significantly higher than that of the CON group (*P* < 0.05). Compared with the MOD group, the kidney index with a loss of 8.05% was observed in the Q7 group, while an increase of 6.9% was found in the ADC group. It was confirmed that *L. plantarum* Q7 treatment could relieve the swelling of the organs significantly (*P* < 0.05).

**Table 2:** Effects of *L. plantarum* Q7 on body weight, organ weight, and visceral Co-efficient in mice.

**Group**	**Initial weight/g**	**Final weight/g**	**Liver weight/g**	**Liver index/%**	**Kidney weight/g**	**Kidney index/%**
CON	20.70 ± 0.82^a^	24.21 ± 1.08^b^	1.04 ± 0.02^a^	4.29 ± 0.22^a^	0.35 ± 0.02^a^	1.47 ± 0.11^a^
MOD	20.54 ± 0.63^a^	23.13 ± 1.13^a^	1.34 ± 0.08^bc^	5.74 ± 0.40^a^	0.41 ± 0.07^b^	1.74 ± 0.27^bc^
Q7	20.71 ± 0.62^a^	25.05 ± 0.72^b^	1.44 ± 0.15^c^	5.74 ± 0.69^a^	0.40 ± 0.02^ab^	1.60 ± 0.12^ab^
ADC	20.79 ± 0.93^a^	21.85 ± 1.15^c^	1.21 ± 0.20^b^	5.56 ± 1.00^b^	0.41 ± 0.03^b^	1.86 ± 0.10^c^

*^a, b, c^Identical letters represent no significant difference and different letters represent significant difference (P < 0.05)*.

The H&E staining showed that HUA caused damage to the viscera of mice, while these pathological features were improved by *L. plantarum* Q7 gavage. As shown in Figure 3, the hepatocytes in the CON group had normal morphology, while it was swollen in the MOD group. The inflammatory cell infiltration was severe, and the fatty vacuole depositions were most obvious in the MOD group, which was alleviated in the Q7 group and the ADC group. On the contrary, the renal tubule lumen was dilated, while the glomerulus was atrophic and deformed in the MOD and ADC groups. The integrant epithelial cells in the MOD and ADC groups displayed edematous and denatured significantly compared with that of the CON group. In contrast, the above adverse symptoms were effectively improved in the Q7 group. The villi in the MOD and ADC groups were swollen and hyperemic. The epithelial cells were exfoliated, and the lymphocytes and plasma cells were infiltrated from the lamina propria. Nevertheless, the length and distribution of villi were recovered, the crypt depth ratios were improved, and the lipid infiltration was reduced in the Q7 group. These findings suggested that *L. plantarum* Q7 might be used as a probiotic to alleviate HUA symptoms.

**Figure 3:** Histopathological analyses of H&E stained liver, kidney sections (×200 magnification), and intense sections (×100 magnification) from mice.

### Regulation of Serum Biochemical Indicators by *L. plantarum* Q7

To examine the effect of *L. plantarum* Q7 on the serum biochemical indicators of HUA mice, supplement with a high purine diet and fructose water and intraperitoneal injection of potassium oxonate were given to mice for 4 weeks. Blood samples were collected for analysis on the 7th, 21st, and 35th day, and the results are shown in Figure 4. It could be seen that after 14 days of modeling, the serum UA level increased to 241.37 ± 14.51 μmol/L, the serum BUN level increased to 13.41 ± 0.54 mmol/L, the serum Cr level increased to 98.73 ± 12.48 μmol/L, and the serum XOD level increased to 2.71 ± 0.24 U/L, which were 1.5 times higher than those of the CON group (*P* < 0.05). Hence, it could be considered that the establishment of HUA models under these experimental methods was successful.

**Figure 4:** Effects of *L. plantarum* Q7 on serum indexes in mice at different time points. **(A)** UA; **(B)** BUN; **(C)** Cr; **(D)** XOD.

After 14 days of *L. plantarum* Q7 gavage, the levels of UA, BUN, Cr, and XOD were significantly decreased compared with the MOD group, while they increased compared with the CON group (*P* < 0.05). The results showed that the levels of UA, BUN, and XOD in the ADC group were all decreased, which were almost equal to the CON group (*P* < 0.05). It was consistent with the report of Wu et al. (21). On the contrary, the Cr level was further increased to 115.74±2.59 μmol/L after giving ALLO. Although ALLO was found to reduce UA by inhibiting uricase activity in the liver (29), Cr was further increased, and weight loss was more severe in the ADC group. A similar phenomenon was observed in organ Co-efficient and H&E pathology. Compared with the CON group, the MOD group and the ADC group exhibited severe injury, whereas the Q7 group achieved remission, which was consistent with the research results of Ni et al. (19). It was suggested that *L. plantarum* Q7 might alleviate HUA by downregulating serum biochemical indicators.

### Elimination of Pro-inflammatory Factors in Mice by *L. plantarum* Q7

It was reported that the pathogenic mechanisms of HUA were associated with the inflammatory response (21). MDA is a common index of peroxidation, and LPS, IL-1β, and TNF-α are important biomarkers of inflammation. The level of these pro-inflammatory factors can reflect the inflammatory response (25). To investigate the correlation between pro-inflammatory and HUA, and provide the scientific basis for the treatment of HUA, the effect of *L. plantarum* Q7 on the pro-inflammatory factors in HUA mice was evaluated. The level of IL-1β and LPS in serum, and the level of IL-1β, TNF-α, and MDA in the homogenate were tested, and the results were shown in Figure 5. These pro-inflammatory factors showed an alarming increase in the MOD group (*P* < 0.05). Compared with the MOD group, the levels of the serum IL-1β and LPS in the Q7 group decreased by 43.05% and 30.73%, respectively (*P* < 0.05), which were better than those of the ADC group and consistent with the CON group.

**Figure 5:** Effects of *L. plantarum* Q7 on the pro-inflammatory factors of mice. **(A)** Serum IL-1β; **(B)** Serum LPS; **(C)** Liver IL-1β; **(D)** Kidney IL-1β; **(E)** Liver TNF-α; **(F)** Kidney TNF-α; **(G)** Liver MDA; **(H)** Kidney MDA.

In the hepatic and nephritic homogenate, the content of IL-1β, TNF-α, and MDA in the MOD group was significantly increased, whereas it decreased after the intervention of *L. plantarum* Q7 (*P* < 0.05). The IL-1β content was reduced by 38.52% and 50.01%, the TNF-α content was reduced by 50.63% and 48.49%, and the MDA content was reduced by 32.44% and 39.10%, respectively (*P* < 0.05). It was confirmed that *L. plantarum* Q7 improved the antioxidant activity, suppressed the abnormalities of pro-inflammatory factors, relieved the inflammation symptoms, as well as ameliorated the occurrence and development of HUA, which was consistent with the study of Wu et al. (21).

### Effect of *L. plantarum* Q7 on UA Metabolism Enzymes and Transporters

The UA is primarily synthesized in the liver, and ADA and XOD are important enzymes involved in UA metabolism. To evaluate the effect of *L. plantarum* Q7 on UA synthesis of mice, the levels of liver ADA and XOD were determined as shown in Figure 6. Compared with the CON group, both ADA and XOD in the liver were significantly increased in the MOD group (*P* < 0.05). Alternatively, the expression levels of ADA and XOD in the Q7 group and ADC group were significantly inhibited. The levels of ADA and XOD were downregulated by 27.82% and 29.41% (*P* < 0.05), which indicated that *L. plantarum* Q7 might reduce the UA level by inhibiting hepatic uric acid synthase.

**Figure 6:** Effects of *L. plantarum* Q7 on metabolism enzyme of mice. **(A)** Liver ADA; **(B)** Liver XOD.

The renal UA excretory transporter NPT1 and the reabsorption transporters GLUT9 and URAT1 played important roles in mediating UA excretion (1, 30). Regulating the expression of NPT1, GLUT9 and URAT1 can effectively keep the balance of the serum UA level, which is an important approach to treat HUA. To demonstrate the effect of *L. plantarum* Q7 on UA excretion of mice, the transporter expression levels of GLUT9, URAT1, and NPT1 involved in UA metabolism were detected. As illustrated in Figure 7, the MOD group had no significant changes in the expression of URAT1 and NPT1 compared with the CON group. However, the level of GLUT9 increased significantly in the MOD group compared with the CON group (*P* < 0.05). Compared with the MOD group, the expressions of reabsorption transporters GLUT9 and URAT1 in the Q7 group decreased by 31.22% and 30.89% (*P* < 0.05), respectively, whereas the expression of excretion transporter NPT1 increased by 45.34% (*P* < 0.05). It suggested that *L. plantarum* Q7 could regulate UA metabolism by reducing reabsorption enzyme and promoting excretion transporter to compensate for UA balance, which was consistent with the reports of Hoque et al. (31), which confirmed that altering transporter expression could regulate UA excretion and thereby ameliorate HUA.

**Figure 7:** Effects of *L. plantarum* Q7 on the transporter expression level of mice.

### Modulation of Gut Microbiota in Mice by *L. plantarum* Q7

Gut microbiota is another crucial factor related to the etiopathogenesis of HUA. It was reported that HUA caused the abnormality in gut microbiota, including a descent in gut microbial diversity and an enrichment in pathogenic bacteria (17). In our previous study, *L. plantarum* Q7 was found to alleviate ulcerative colitis by altering intestinal flora (23). In this study, we explored whether it could regulate the intestinal flora of HUA mice. The effect of *L. plantarum* Q7 on intestinal microbiota of HUA mice was performed by Miseq sequencing analysis of 16S rRNA. It was found that the microbial richness, evenness, and diversity were significantly decreased in the MOD group in comparison with those of the CON group. *L. plantarum* Q7 treatment could moderately restore the species diversity, richness, and community evenness (Figure 8A).

**Figure 8:** Effects of *L. plantarum* Q7 on gut microbe of mice. **(A)** α-diversity indexes calculated with QIIME2 according to ASV/OTU numbers of each group (*P* < 0.05). **(B,C)** Venn diagram of ASV/OTU in the feces. **(D)** β-diversity evaluated using the weighted UniFrac-based PCA. **(E)** β-diversity evaluated using the weighted UniFrac-based PCoA. **(F)** Bar graphs showing the relative abundance of different bacteria at the phylum level. **(G)** Bar graphs showing the relative abundance of different bacteria at the gene level. **(H)** Correlation matrix between the microbiota and inflammatory cytokines. **(I)** Changes of the Bac/Firm Ratio in the different groups (*P* < 0.05).

The composition information of species in each group was used to display in the Venn diagram. It was observed that 3,071 OTUs overlapped in the CON, MOD, and Q7 groups, 1,127 OTUs were present in both the CON and MOD groups, 1,294 OTUs were present in the MOD and Q7 groups, and 2,760 OTUs were present in the CON and Q7 groups, which were higher than those of the ADC group (Figures 8B,C). Compared with the MOD group, intestinal microbial composition in the Q7 group was more similar to the CON group (Figures 8D,E). The results showed that the gut flora of the MOD group was significantly different from that of the CON group, which could alleviate the shift by *L. plantarum* Q7 gavage.

Compared with the CON group, the composition of gut microbiota at the phylum level showed that the relative abundance of *Firmicutes* was significantly decreased, whereas *Bacteroidetes* and *Proteobacteria* were markedly increased in the MOD group (Figure 8F). This imbalance of gut microbiota was recovered in the Q7 group, and the corresponding symptoms of HUA were further relieved, which was consistent with the reports of Zhao et al. (32). The difference of gut microbiota in each group at the genus level suggested that the relative abundance of *Muribaculaceae* was increased after HUA modeling, the relative abundance of *Lachnospiraceae*_NK4A136_group, *Prevotellaceae*_UCG-001 and *Prevotellaceae*_NK3B31_group were decreased, while those flora in the Q7 group were recovered to the level of CON group (Figure 8G). In addition, *Akkermansia*, a promising probiotic (33, 34) was increased significantly in the Q7 group, suggesting that *L. plantarum* Q7 could improve the intestinal flora disorder of HUA mice. Although it was confirmed that *L. plantarum* Q7 could regulate intestinal microbiota and alleviate HUA, the specific functional components and the exact mechanism remained to be explored.

Other studies have found that HUA caused the increase of inflammatory factors (21, 27), such as IL-1β, TNF-α, LPS, and MDA, which indicated HUA could be relieved by regulating inflammation. The relationship between the intestinal flora and inflammatory cytokines was conducted by correlation analysis. It could be discovered that *Bacteroidetes* and *Deferribacteres* were positively correlated with inflammatory cytokines, while *Firmicutes* and *Chloroflexi* were negatively correlated with inflammatory cytokines (Figure 8H). Furthermore, the ratio of *Bacteroidetes* to *Firmicutes* (Bac/Firm ratio) was recovered nearly to the level of the CON group by *L. plantarum* Q7 therapy (Figure 8I), which suggested that *L. plantarum* Q7 could shape the intestinal microbiota of the HUA mice. The results indicated that there was a certain correlation among HUA, inflammatory factors, and intestinal flora, while the specific mechanism remained to be studied further.

## Conclusion

The UA-lowering activity of *L. plantarum* Q7 was investigated *in vitro* and *in vivo*. *L. plantarum* Q7 exhibited excellent capability to regulate UA metabolism and alleviated HUA in the mice models. It was observed that *L. plantarum* Q7 could downregulate the serum biochemical indexes, restore the organ injury, and regulate the UA metabolism enzyme and transporter expression. Moreover, an inseparable relationship between the intestinal flora and HUA was found. *L. plantarum* Q7 could improve the imbalance of gut microbiota and suppress inflammation. These findings highlighted that *L. plantarum* Q7 might alleviate HUA by reshaping intestinal flora.

## Data Availability Statement

The datasets presented in this study can be found in online repositories. The names of the repository/repositories and accession number(s) can be found in the article/supplementary material.

## Ethics Statement

The animal study was reviewed and approved by SPXY2022011201.

## Author Contributions

HY: conceptualization, project administration, supervision, funding acquisition, and writing, reviewing, and editing. JC, YB, and TW: formal analysis. JC and HH: software. JC and YB: data curation. JC, YB, and HH: methodology and writing the original draft. QL and YL: visualization. All authors contributed to the article and approved the submitted version.

## Funding

This study was supported by the National Natural Science Foundation of China (Nos. 32172180 and 31771988).

## Conflict of Interest

The authors declare that the research was conducted in the absence of any commercial or financial relationships that could be construed as a potential conflict of interest.

## Publisher's Note

All claims expressed in this article are solely those of the authors and do not necessarily represent those of their affiliated organizations, or those of the publisher, the editors and the reviewers. Any product that may be evaluated in this article, or claim that may be made by its manufacturer, is not guaranteed or endorsed by the publisher.
